# The Impact of COVID-19 Outbreak on CO_2_ Emissions in the Ten Countries with the Highest Carbon Dioxide Emissions

**DOI:** 10.1155/2023/4605206

**Published:** 2023-06-13

**Authors:** Marzieh Ronaghi, Eric Scorsone

**Affiliations:** Department of Agricultural Food and Resource Economics, Michigan State University, East Lansing, USA

## Abstract

The environmental pollution during the COVID-19 crisis has declined dramatically due to quarantines that have severely reduced transport and industry but has had little effect on the steady rise in CO_2_ concentrations in the atmosphere. Through the Paris Agreement, countries are working to reduce the emissions of these pollutants, for example, by burning fossil fuels. These greenhouse gases trap heat near the earth's surface and raise the temperature. This global warming threatens global food resources. In times of corona crisis and environmental pollution, especially in countries with the highest CO_2_ emissions, governance is a key factor that explains the poor economic, social, and environmental performance of many countries. Governance plays an important role in controlling these crises. In this study, the World Bank's governance indicators have been used to examine the relationship between governance and economic performance and its impact on CO_2_ emissions during the COVID-19 outbreak period. Also, the Tobit panel model with a limited-dependent model from 2011 to 2020 has been used. Several economic factors and governance variables are also considered. Given the negative relationship between governance and CO_2_ emissions during the COVID-19 outbreak, the role of governance in reducing environmental pollution is emphasized, and it is shown that policymakers can take appropriate measures by implementing good governance and enforcing the right laws to control the corona epidemic and also reduce carbon emissions in the long run.

## 1. Introduction

The global crisis caused by the COVID-19 epidemic has led to an unprecedented reduction in daily carbon dioxide emissions. Although there is no real-time measure of carbon dioxide emissions and emissions are usually reported annually, scientists have been able to estimate changes in emissions using information on energy consumption, economic activity, and other factors. A study published in Nature Climate Change estimated a reduction of 17% in daily emissions in early April 2020 (Figure 1). Greenhouse gas emissions had a reduction of 17 percent from a year earlier on April 7. At the time, China, the United States, India, and other major carbon-emitting countries were all at high levels of quarantine. Overall, daily carbon dioxide emissions decreased by an average of 8.6% between January and April compared to the same period in 2019 (Figure 1). However, the full impact on the annual emission in 2020 depended on the trend and evolution of quarantine and disease control measures and the final speed of economic recovery [1].

In the short term, carbon dioxide emissions usually increase and decrease at the same time as economic activity. This means that there is a very strong correlation between real gross domestic production (GDP) growth and emissions [2]. For example, during the financial crisis of 2008 and the ensuing recession, global GDP fell by 1.5% and global emissions also decreased by 1.3% (Figure 2). Due to the sharp decline in global economic growth caused by the epidemic, greenhouse gas emissions have declined similarly [3]. As shown in Figure 2, the coronavirus can cause the largest annual reduction in carbon dioxide emissions. Precrisis GDP estimates show that carbon dioxide will increase by more than 1% by 2020 (470 million tonnes of CO_2_).

The reduction in emissions due to the pandemic could be greater than that would be expected from a more normal recession. The reduction in carbon dioxide emissions from the epidemic is expected to be large, not only because of the magnitude of the impact on global growth but also because of the sectors that have been particularly affected [4]. The epidemic has led to a significant reduction in economic activity, including exports and imports around the world, due to a sharp decline in transportation and production. The airline industry suffered a severe blow as a growing number of countries imposed travel restrictions. Electricity generation, transportation, and industrial activities account for more than 80% of carbon dioxide emissions from fuel combustion [5]. This means that the reduction in greenhouse gas emissions could be more than a normal recession because the energy-consuming sectors were severely affected and also caused a reduction in foreign investment. With millions of people at home, all industrial sectors were shut down. Manufacturers, meanwhile, have halted coal mining, a key activity in CO_2_ emissions, in response to a weak market due to the corona outbreak that has infected some workers. Also, domestic travel and air travel decreased, and in this regard, exports and imports in countries also decreased [6]. During this period, according to government statements, a large number of employees lost their jobs or worked remotely, leading to a reduction in GDP, so this had a clear effect on carbon dioxide emissions (U.S. Bureau of Labor Statistics, 2022).

While much attention has been paid to the unprecedented reduction in emissions, it is important to keep in mind that it is not the emission of greenhouse gases, but their reserves, that is, the concentration of greenhouse gases in the atmosphere that leads to climate change. Climate change is a cumulative problem because greenhouse gases accumulate in the atmosphere over time. The dramatic reduction in carbon dioxide emissions resulting from the coronavirus epidemic means that the flow that contributes to the concentration of carbon dioxide in the atmosphere is reduced but no decrease in atmospheric carbon dioxide is observed.  Figure 3 shows that China and the United States are the world's largest polluters with emissions of 10.6 and 4.7 billion tons of carbon dioxide by 2020. Despite being the second largest polluter in the United States, US greenhouse gas emissions have dropped 16 percent since 2010. In comparison, China's carbon dioxide emissions have increased by almost 25%. In fact, the concentration of carbon dioxide in the atmosphere reached about 418 parts per million in May 2020, which was the highest level ever recorded [7]. In addition, the decline in emissions observed is likely to be reversed as quarantines are lifted and economies return to growth. This was the case in previous recessions, while greenhouse gas emissions fell by 1.3% during the Great Depression in 2009, they increased by almost 6% in 2010, bringing CO_2_ concentrations back to prerecession [1].

Switching to technologies with lower CO_2_ emissions, along with investing in strategies to reduce existing carbon dioxide concentrations in the atmosphere, can have a more lasting impact on reducing climate change. In addition, the reduction in greenhouse gas emissions obtained in this way is likely to impose less difficulty in comparison to the economic pain due to severe short-term reductions, such as those of the current recession and quarantine policies (TeRC, 2022).

The fact that large reductions in emissions as a result of painful and dramatic conditions such as the recession and quarantine do not significantly alter CO_2_ concentrations suggests that active policies are essential. It is the time now to design crisis recovery policies that include the growth of the economy. According to new research, “green recovery” could help reduce 0.3°C in the path of global warming. Active decarbonization policies, as well as the reduction of other greenhouse gases around the world, are needed to reduce the risk of the next global climate crisis. Therefore, in recent years, special attention has been paid to the governance of countries to adopt policies to reduce greenhouse gases [8].

Global Environmental Governance (GEG) is a set of organizations, policy instruments, funding mechanisms, laws, procedures, and norms that govern global environmental protection processes [9].

Protecting the environment and the rights of future generations is one of the most important responsibilities of the government, civil society, and private sector [10–12]. Because environmental pollution affects the whole society, governance indicators play an important role in controlling environmental pollution by influencing environmental and social policies. Especially during the outbreak of COVID-19, many countries with the highest levels of CO_2_ were affected by this disease (Figure 4) and had a high ranking in the number of patients with the COVID-19 disease. Implementing good governance in countries has led to successful disease control.

Given the important role of good governance in economic, social, and political performance, as well as its impact on reducing environmental pollution, improving governance components such as Regulatory Quality, civil liberties, and public participation in environmental protection directly improves the quality of the environment in a country [13, 14]. Since governance has a significant impact on all areas of a country, the establishment of good governance makes the government more efficient in adopting sustainable policies and environmental protection [15]. Therefore, by improving the indicators of good governance, including the adoption of appropriate and sustainable policies, the implementation of appropriate laws, deterrence of violators of the law, and compliance with standards, environmental pollution in the country will be reduced [16].

In terms of controlling the corona crisis as well as controlling environmental pollution, especially in the countries with the highest CO_2_ emissions, the role of governance has become much more highlighted than before. While several studies have examined the effects of economic and regulatory factors on CO_2_ emissions [15, 17–20] (Nchofoung 2022; Latifi et al. 2021), none of these studies have focused on the effect of corona outbreaks on CO_2_ emissions along with economic and Regulatory Quality factors. Given the environmental pollution in countries with the highest CO_2_ emissions and also the vital role of governance in explaining environmental pollution, the present study focuses on the impact of corona outbreaks on CO_2_ emissions and economic and governance factors in these countries.

## 2. Literature Review

Greenhouse gases, including CO_2_ emissions, are rising rapidly, and the earth's climate is constantly warming [21–24]. However, knowledge about the comprehensive role of the terrestrial biosphere on a regional to global scale under climate change is still limited [25, 26]. This is an opportunity for everyone, including policymakers, to develop and implement strategies to reduce greenhouse gas emissions, including CO_2_, one of the fastest growing greenhouse gases. This is a great time to learn the strategies of nonlockdown measures implemented during COVID-19 and their implementation to curb global carbon emissions and reduce the impact of climate change in the long run [27].

Recent research on the environmental impact of COVID-19 during the 2020s and pre-COVID-19 periods has been conducted for a relatively short period of time (weeks to months of COVID-19 and non-COVID-19 periods). However, these studies may include the effects of activities not directly related to COVID-19, such as meteorological and seasonal conditions, which may not be the same in two different years during the same period as well as in two different geographical locations. For example, Liu et al. [28] found that the first months of 2020 were extremely hot in most of the Northern Hemisphere compared to the same period in 2019, resulting in lower CO_2_ emissions in 2020 than in 2019 when there were no external forces such as COVID-19. In addition, COVID-19 quarantine measures can have indirect positive and negative effects on the environment.

Another study in the corona period (Monserrate et al. 2020) [14, 29] focused on China, the United States, Italy, and Spain dealing with the indirect positive and negative effects of the COVID-19 epidemic on the environment. While significant correlations were found between air quality improvement and quarantine measures, they also noted the indirect negative effects of reduced waste recycling. Increased waste and land and climate pollution during quarantine measures has shown that the reduction in greenhouse gas emissions currently observed in some countries is only temporary and a significant increase in emissions after the end of the epidemic or the abolition of quarantine measures will be possible [30, 31].

Friedlingstein et al. [32] also studied the impact of COVID-19 quarantine on various sectors. They showed that at the peak of COVID-19 in April, the areas responsible for about 90% of global fossil CO_2_ emissions were at a limited level. CO_2_ emissions in aviation fell by 75%, surface transport by 50%, electricity generation by 15%, and industry by 35%. The reduction in CO_2_ emissions had no noticeable effect on atmospheric CO_2_ or climate change. The reduction in accumulated greenhouse gas emissions so far is very small compared to the reduction in greenhouse gas emissions needed to counter the climate change. Changes in active mobility in large cities in response to a crisis can be partially permanent with many benefits.

In another similar study, Yadav et al. (2020) found that responses to COVID-19 led to an unintended reduction in carbon dioxide (CO_2_) emissions across the city, which reduced CO_2_ emissions in Los Angeles and Washington DC/Baltimore during March and April 2020 with three lines of evidence using methods that are increasingly dependent on the model, including an inverse model for estimating relative emission changes in 2020 compared to 2018 and 2019. The decline in March (25 percent) in Washington DC/Baltimore was largely due to lower natural gas consumption associated with a hot spring, while the decline in April (33 percent) was associated with changes in gasoline sales. In contrast, only a fraction of the March (17%) and April (34%) decline in Los Angeles was explained by traffic congestion. The methods and measurements used in this paper provide the benefits of atmospheric CO_2_ observations to provide timely insights into changing rapid emission patterns that can empower cities to effectively correct CO_2_ reduction activities.

In addition, Drudi [33] analyzed the consequences of climate change for the implementation of monetary policy in the Eurozone. Weather as well as the regulatory and financial effects of reducing carbon emissions was examined. In this regard, they assessed the need to adapt macroeconomic models and the economic forecasts of Eurosystem/ECB staff in monetary policy decisions. They also considered the consequences of climate change for monetary policy implementation, in particular the consequences of monetary policy transitions, natural interest rates, and the correct identification of shocks. Their model simulations using the New Area-Wide Model of the euro area (NAWM) show how climate change interactions and financial failures can significantly limit the ability of monetary policy to respond to standard business cycle fluctuations. Their paper was in line with the European Central Bank's mandate, analyzing a set of potential monetary policy measures to address climate risks.

Burck and Uhlich [34] evaluated the Climate Change Performance Index; the results show that monitoring climate reduction efforts in 60 countries plus the European Union account for 92% of global greenhouse gas emissions. It is important to note that the Climate Change Performance Index (CCPI) is calculated using only production-based publications. The CCPI, therefore, follows the current practice of national emissions accounting and follows the logic that the country that produces these pollutants is also responsible. In addition, they showed that it is important to note that more than half of the CCPI rating indicators are qualified in relative terms (better/worse) rather than absolute. So, even high-ranking countries have no reason to sit still. On the contrary, the results show that even if all countries are as committed as the current leading countries, efforts to prevent dangerous climate change will not be enough.

Recent studies on the effects of COVID-19-related activities on air pollutants and greenhouse gas emissions used data from weeks to months on a local to global scale. In general, the importance and consequences of quarantine measures are not yet well understood [30, 35]. To the best of researchers' knowledge, no study has examined the impact of economic activity during the COVID-19 era on CO_2_ emissions using annual observations due to data shortages. Annual carbon dioxide emission data are essential to investigate the combined effects of COVID-19-related activities. Since this large amount of data has only recently become available by 2020, this study examines the effects of the COVID-19 epidemic on global carbon dioxide emissions from 2011 to 2020, focusing on ten countries with the highest CO_2_ emissions and COVID-19 patients. Therefore, the main objectives of this study are (1) to investigate the effects of quarantine measures due to COVID-19 epidemic on annual CO_2_ emissions and (2) study annual carbon emissions at global levels in ten countries with the highest annual CO_2_ emissions and COVID-19 patients.

## 3. Methodological Approach

CO_2_ emission is one of the serious environmental crises in human life. Many studies have investigated the effects of various factors on CO_2_ emissions [36, 37]. During the COVID-19 outbreak, carbon dioxide emissions were reduced due to quarantine in many countries.

This research uses the Panel Tobit model following Bruno [38]; Busse and Bernard [39]; and Chang et al. [40]. In a Panel Tobit model, individual-specific and time-invariant effects are modelled as random effects; a fixed effects model is plagued by the incidental parameter problem. However, in data-censoring applications under the maintained assumption (*H*0: *ξ*) = 0, adding $\bar{X}$*i* to the random effects Tobit model solves the unobserved heterogeneity problem.

(1) $$\begin{array}{c} Y_{it}={\beta X}_{it}+C_{i}+u_{it}\;t=1,2,\ldots \ldots ,T\text{,}\\ C_{i}=\psi +{\overset{̿}{X}}_{i}\bar{\xi }+\alpha_{i}\text{,} \end{array}$$

where *C*_*i*_ is the unobserved effect and *Xi* contains *X*_*it*_ for all *t*. These equations represent a data-censoring model, and *β* is of primary interest.

In this paper, we use panel data with a limited dependent variable (LDV). According to the Tobit method, we must define a threshold where the data under that threshold are censored (considered as zero values) and the data above it are visible. The 10 countries are considered with the highest CO_2_ emissions; among them, the countries that are also in the list of ten countries with the highest corona cases have *Y* greater than zero and the rest are considered zero on the list.

According to the studies reviewed in the literature review section, the most important economic variables affecting CO_2_ emissions are GDP growth, exports, imports, foreign direct investment, and governance. Due to the importance of trade impacts on environmental pollution, the choice of exports and imports is emphasized in the literature [41, 42].

### 3.1. The Panel Tobit Model

LDV models are characterized by the presence of lagged-dependent variables and serially correlated errors. In the panel Tobit model structure, the conventional estimation methods used for simple panel data models do not apply to the Tobit panel model due to our use of time-dummy variables and lagged dependent variables.

To maximize the corresponding likelihood function and specify the conditional error distribution, random effects can also be used. The random effect approach allows time-dummy variables, time-varying and time-invariant. In addition, identification is typically simple assuming distributed errors.

The structure of the Tobit panel econometric model is [38]

(2) $$\begin{array}{c} y_{it}^{*}=\beta^{\prime }x_{it}+u_{it},\;i=1,2,\ldots \ldots ,N\;t=1,2,\ldots ..,T\text{,} \end{array}$$

(3) $$\begin{array}{c} u_{it}=v_{i}+\varepsilon_{it}\;\left(v_{i}∼NID\left(0,\sigma_{v}^{2}\right)\right)\;\left(\varepsilon_{it}∼\;NID\left(0,\sigma_{\varepsilon }^{2}\right)\right)\text{,} \end{array}$$

where the observed variables are

(4) $$\begin{array}{c} y_{it}=\left\{\begin{array}{ll} y_{it}^{*}\text{,} & if\;y_{it}^{*}>0\text{,}\\ 0\text{,} & otherwise\text{,} \end{array}\right. \end{array}$$

where *y* is a dual dependent variable and *x* is an independent variable. The common error term, u_it_ in equation (3), is correlated with time. The error component model splits u_it_ into a time-invariant individual random effect (RE), *v*_*i*_, and a time-varying idiosyncratic random error, *ε*_it_.

If the *ν*'s and the *Ɛ*'s are independent and *d*_it_ = 1 for uncensored observations and *d*_it_ = 0 for censored observations, the likelihood function for each individual, marginalized with respect to the random effect *v*_*i*_ is as follows:

(5) $$\begin{array}{c} l_{it}=\int_{-\infty }^{\infty }{\left[\frac{1}{\sigma_{\varepsilon }}\emptyset \left(\frac{y_{it}-{\beta^{\prime }x}_{it}+vi}{\sigma_{\varepsilon }}\right)\right]}^{d_{it}}.\;{\left[\Phi \left(\frac{-{\beta^{\prime }x}_{it}+vi}{\sigma_{\varepsilon }}\right)\right]}^{\left(1-d_{it}\right)}f\left(vi,\sigma_{i}\right)dvi\text{,} \end{array}$$

where ∅ (.) is the probability density function, Φ (·) is the cumulative distribution function of the standard normal distribution, and f(*v*_*i*_, *σ*_*i*_) is the normal density with mean *v*_*i*_ and standard deviation *σ*_*i*_. For *T*_i_ observations, the likelihood function is

(6) $$\begin{array}{c} L_{it}=\int_{-\infty }^{\infty }\overset{t=T_{i}}{\underset{t=1}{\prod }}.{\left[\frac{1}{\sigma_{\varepsilon }}\emptyset \left(\frac{y_{it}-{\beta^{\prime }x}_{it}+vi}{\sigma_{\varepsilon }}\right)\right]}^{d_{it}}.{\left[\Phi \left(\frac{-{\beta^{\prime }x}_{it}+vi}{\sigma_{\varepsilon }}\right)\right]}^{\left(1-d_{it}\right)}f\left(vi,\sigma_{i}\right)dvi\text{,} \end{array}$$

The dependent variable is CO_2_ in this research. The independent variables are GDP growth, exports, imports, foreign direct investment, and governance. All independent variables are chosen based on the Wald test and the Lm test with a significance level of 5%. Thus, all the included independent variables add significant explanatory power to the model, and removing any one substantially reduces the model's fit. The hypothesis of random effects is not rejected by the Breusch–Pagan test, so the empirical model is as follows [43]:

(7) $$\begin{array}{c} {Co2}_{it}=\left\{\begin{array}{ll} {Co2}_{it}^{*}\text{,} & if\;y_{it}^{*}>0\text{,}\\ 0\text{,} & other\;wise\text{,} \end{array}\right.\\ y_{it}^{*}=\beta^{\prime }{GDP}_{it}+\beta^{\prime }E_{it}+\beta^{\prime }M_{it}+\beta^{\prime }{GOV}_{it}+\beta^{\prime }F_{it}+u_{it}\text{, }i=1,2,\ldots \ldots ,N\;t=1,2,\ldots \ldots ,T\text{,}\\ U_{it}=v_{i}+\varepsilon_{it}\left(v_{i}∼NID\left(0,\sigma_{v}^{2}\right)\right)\left(\varepsilon_{it}∼\;NID\left(0,\sigma_{\varepsilon }^{2}\right)\right)\text{,}\\ l_{it}=\int_{-\infty }^{\infty }{\left[\frac{1}{\sigma_{\varepsilon }}\emptyset \left(\frac{y_{it}-\beta^{\prime }{GDP}_{it}-\beta^{\prime }E_{it}-\beta^{\prime }M_{it}-\beta^{\prime }{GOV}_{it}-\beta^{\prime }F_{it}+vi}{\sigma_{\varepsilon }}\right)\right]}^{d_{it}}.\;{\left[\Phi \left(\frac{-\beta^{\prime }{GDP}_{it}-\beta^{\prime }E_{it}-\beta^{\prime }M_{it}-\beta^{\prime }{GOV}_{it}-\beta^{\prime }F_{it}+vi}{\sigma_{\varepsilon }}\right)\right]}^{\left(1-d_{it}\right)}f\left(vi,\sigma_{i}\right)dvi\text{.} \end{array}$$

The sample likelihood function is the product of *L*_*i*_ over the *N* individuals:

(8) $$\begin{array}{c} L=\overset{N}{\underset{i=1}{\sum }}\ln\;\left(l_{i}\right)\text{.} \end{array}$$

Equation (8) does not become a sum because the integral is a product. Interrelationships between observations prevent the division of the probability share of T*i* periods for individual *i* when there is a serial correlation. When the number of time periods is more than three or four, classical estimation methods are impossible in a T-dimensional integral. In this research, maximum likelihood estimation for limited dependent variable panel data is available for a simple random disturbance structure, and we use STATA for Tobit panel models. The random effects model estimation assumes that *ε* is serially uncorrelated, *v*_*i*_ are uncorrelated across individuals, and *v*_*i*_VI *x*_*i*_∼NID (0, *σ*^2^).

## 4. Data Description and Analyses

This study covers annual data for 2011–2020 for a group of countries that have the highest CO_2_ emissions and corona cases. Panel data are a collection of data by a large number of cross-sectional variables (*N*) over a period of time (*T*). Characteristics of panel data include the following: they show heterogeneity, provide greater degrees of freedom and more diversity in data, provide less correlation between variables, and thus produce a more efficient estimator [44]. Panel data allow the individual to have the power of cross-sectional analysis and time series. Not only can we see how the cross-sectional units change over time but we can also see the difference between the cross-sectional units. In addition, all available data are used, and as a result, observation errors are reduced [45]. The descriptive statistics of the variables are shown in Table 1.

First, we used Fisher's generalized unit root to perform stationary tests [46]. In the Fisher test for panel data, the null hypothesis of a unit root is rejected at the 5% level of significance (Table 2).

The cross-section correlation test is performed using the freeze test (Table 2). The null hypothesis of no correlation was rejected at the 5% level of significance. We also use the Hausman test to examine fixed versus random effects. The null hypothesis of no fixed effects is accepted (Table 3), so the random effects model is used.

## 5. Estimation Results

In this study, the effects of economic factors and governance index on CO_2_ emissions are estimated with the Tobit panel model during the COVID-19 outbreak and the results are presented in Table 4.

The good governance index has a significant negative effect on CO_2_ emissions (Table 4). Improving each of the governance indicators, such as the regulatory quality index, improves the quality of the country's environment [13]. Therefore, good governance has a great impact on controlling air pollution and also controlling the coronavirus. Good governance plays an important role in the sustainability of environmental policies. Environmental governance regulates the global environmental protection and includes organizations, funding mechanisms, procedures, and norms. The goal of global environmental policies is to improve the state of the environment and ultimately sustainable development [47]. In the Tobit panel method, the coefficients must be converted in order to determine the elasticities. The total elasticity is the effect of one percentage change in *x* on *y*. The elasticity of the governance is −0.23. It has the largest elasticity for CO_2_ emissions found in this study (Table 5). This means that if the amount of the governance increases by one percent, the CO_2_ emissions will decrease by 0.23 percent. Due to the large elasticity of the governance, the important role of governance was shown in both environmental pollution reduction policies and corona outbreak control policies in this study.

GDP growth has a positive relationship with increasing environmental pollution and increasing carbon dioxide emissions (Table 4). The elasticity of GDP is 0.02 with a positive sign. This elasticity shows that if GDP increases one percent, CO_2_ emissions increase by 0.02 percent, assuming other factors are constant (Table 5). With the growth of GDP, production has increased in many parts of the country and the increase in production is accompanied by increased use of natural resources, energy, and various fuels and leading to increased emissions of various environmental pollutants such as CO_2_ emissions [48]. These results indicate more pollution in the countries with richer economies. As mentioned above, due to the direct relationship between GDP and environmental pollution, carbon dioxide emissions decreased during the COVID-19 outbreak due to reduced production.

Increased exports significantly increase CO_2_ emissions (Table 4). Puliafito et al. [49] in their study concluded that increasing exports stimulates more production and use of food preservatives in the food industry, artificial colors, and more modern packaging and plastic containers. All of these activities led to more energy utilization and increased CO_2_ emissions. In addition, exports require fuel for transportation, both by air and by land, and increase environmental pollution [50]. The elasticity of export is 0.07 with a positive sign. This elasticity shows that if exports increase one percent, CO_2_ emissions increase by 0.07 percent, assuming all other factors are stable (Table 5). Tunc et al. [6] also showed that increased exports are associated with increased CO_2_ emissions. As noted, due to the direct link between exports and environmental pollution, declining exports due to reduced transport led to carbon dioxide emissions during the COVID-19 outbreak.

Unlike exports, imports reduce production. Reducing production by reducing energy and fuel consumption leads to reduced carbon dioxide emissions. This finding is similar to the results of a study by Faizi et al. [51].

Increasing foreign direct investment indirectly increases environmental pollution (Table 4). Because foreign investment is accompanied by greater economic growth and technology transfer, the introduction of new processes to increase management skills [52] leads to increased production and emissions of carbon dioxide. Because higher levels of economic activity (production and consumption) are associated with increased use of energy and raw materials, it therefore increases CO_2_ emissions. The elasticity of FDI is 0.02 with a positive sign. This elasticity shows that if FDI increases by one percent, CO_2_ emissions increase by 0.02 percent, assuming all other factors are stable (Table 5). The decline in foreign investment during the corona outbreak reduced the production and emissions of carbon dioxide.

The rho is 0.99. It shows that 99% of the variance is due to differences across panels. “rho” is known as the intraclass correlation.

(9) $$\begin{array}{c} Sigma\;u=sd\;of\;residuals\;within\;groups\;ui\text{,}\\ Sigma\;e=sd\;of\;residuals\;\left(overall\;error\;term\right)\;ei\text{,}\\ Rho=\frac{{\left(sigma\;u\right)}^{2}}{{\left(sigma\;u\right)}^{2}+{\left(sigma\;e\right)}^{2}}\text{.} \end{array}$$

Table 5 shows the elasticities for all variables. As shown in Table 5, these elasticities are small relative to the elasticities for governance. It is clear that governance plays a very important role in controlling environmental pollution and adopting appropriate policies to reduce air pollution in countries with the highest levels of carbon dioxide emissions.

## 6. Conclusions

Today's world is facing a series of social and environmental crises. One of the most dangerous crises in recent years has been the outbreak of the coronavirus, which has reduced the environmental pollution crisis due to quarantine in many countries. The corona outbreak crisis has for some time been able to reduce the emission of pollutants and greenhouse gases that pose a serious threat to human life on Earth [53].

This research is in line with several recent studies on how quarantine measures significantly affect carbon emissions in the short term. Although the reduction in carbon emissions was temporary, it showed that if good governance with proper regulation in the city, country, continent, and world levels could be achieved, we could reduce carbon emissions in the long run.

This study examined several large countries with the highest carbon emissions and evaluated the impact of several economic factors and governance indicators on carbon dioxide emissions in each country. Long-term quarantine measures will significantly reduce carbon emissions by 2020. In contrast, several large countries were either slightly affected by COVID-19 or did not take strict quarantine measures and had little or no impact on carbon emissions in 2020 compared to 2019. As a result, this study agrees with Hale and Leduce that a significant reduction in carbon emissions is possible only with fundamental and lasting changes in human activity in the long run [54, 55]. However, given the negative relationship between governance and CO_2_ emissions, an important finding from this study during the COVID-19 outbreak could help policymakers implement good governance and strengthen governance indicators such as quality of regulation by enforcing proper laws and taking the right steps to reduce carbon emissions in the long run.

This study does not determine the amount of real carbon emissions into the atmosphere. However, this study quantifies the overall impact of economic activity and governance index associated with the COVID-19 epidemic on carbon emissions in several environmentally polluting countries. In the future, comparing carbon emissions for quarterly and six-month periods is recommended to quantify changes in carbon emissions in the years before, in, and after COVID-19. In addition, it is recommended that all types, lengths, and degrees of measures taken during the epidemic be considered to compare carbon emissions in large cities and countries.

Also, in the corona era, it is better to pay more attention to environmental studies in the countries with the highest carbon dioxide emissions in order to adopt appropriate policies to reduce environmental pollution, inspired by the corona conditions in the future.

## Figures and Tables

**Figure 1:** Daily Global CO_2_ Emissions (1960–2020)

**Figure 2:** Precrisis GDP estimates suggested that CO_2_ would rise by more than 1% in 2020 (470 Mt CO_2_).

**Figure 3:** Carbon dioxide emissions (million metric tons) in 2020, by selected 10 countries with the highest CO_2_ emissions.

**Figure 4:** Daily new confirmed COVID-19 cases per million people in 2020–2022.

**Table 1:** The descriptive statistics of model variables.

Variable	Maximum	Minimum	Standard deviation	Mean
CO_2_ emissions (metric tons per capita)	17.69	1.40	4.74	9.01
Governance	1.82	−1.52	0.95	0.28
GDP growth	13.93	−15.67	4.03	2.99
Export	23.63	0.06	6.41	4.54
Import	3.98	−0.01	0.87	1.45
FDI	52.22	13.24	9.07	25.29

**Table 2:** The Fisher unit root test results and freeze test.

Method	Value	*P* value
Chi-square and Fisher Dickey Fuller	36.32	0.01
Freeze cross-section correlation	86.04	0.02

**Table 3:** Hausman test results.

Hausman Test	Value	*P* value
Re	12.32	0.46

Notes: Breusch–Pagan test probability distribution *P*=0/00.

**Table 4:** The results of the Tobit panel.

Variables	Coefficient estimates	*Z* statistics	Standard deviation estimates	*P* value
Governance	−0.25^*∗∗∗*^	−3.12	0.08	0.03
GDP growth	0.02^*∗∗*^	2.86	0.007	0.00
Export	0.06^*∗∗∗*^	3.01	0.02	0.01
Import	−0.04^*∗*^	−1.95	0.02	0.05
FDI	0.01^*∗∗*^	2.51	0.004	0.02
Sigma *u*	4.81^*∗∗∗*^	4.15	1.16	0.00
Sigma *e*	0.41^*∗∗∗*^	13.23	0.03	0.00
Rho	0.99		0.003	

Notes: ^*∗*^, ^*∗∗*^, and ^*∗∗∗*^ denote statistical significance at the 10%, 5%, and 1% levels, respectively.

**Table 5:** Elasticity frequency of independent variable.

Variable	Total elasticity	*Z* statistics	Standard deviation estimates
Governance	−0.23^*∗∗*^	−2.86	0.08
GDP growth	0.02^*∗∗*^	2.23	0.009
Export	0.07^*∗∗*^	2.34	0.03
Import	−0.04^*∗*^	−1.98	0.02
FDI	0.02^*∗∗∗*^	3.98	0.005

Notes: ^*∗*^, ^*∗∗*^, and ^*∗∗∗*^ denote statistical significance at the 10%, 5%, and 1% levels, respectively.

## Data Availability

The data used to support this study are available at https://data.worldbank.org/.
